# A Comprehensive Evaluation Method for the Effectiveness of Public Health-Oriented Music Performance Art Based on Blockchain Technology

**DOI:** 10.1155/2022/8307291

**Published:** 2022-09-14

**Authors:** Yiran Shang

**Affiliations:** Institute of Art and Design, Changsha University of Science & Technology, Changsha, Hunan 410114, China

## Abstract

Music can promote the development of physical and mental health, and its therapeutic utility has begun to receive widespread attention from scholars, who have systematically studied the therapeutic methods, processes, and utility of music with the theme of music therapy, and the topic has been extended from music therapy at the individual level to the public health domain. Therefore, it is worthwhile to further explore how the effectiveness of music as a performing arts activity in the public health domain is evaluated. However, most of the current studies focus on the evaluation of the effects of music on individual physical and mental health, and few involve the evaluation of music performing arts activities in the public health domain, which greatly hinders the potential of music performing arts applications in the public health domain. Therefore, this study proposes a dynamic and comprehensive evaluation scheme based on the cross-chain technology in blockchain and establishes a cross-chain-based information exchange model for the feasibility of information exchange between music performing arts and public health. The research findings can not only provide theoretical guidance for the formulation of public health policies but also provide technical support for the comprehensive evaluation of the effectiveness of music performing arts activities.

## 1. Introduction

In recent years, with the development of society and the deepening of the aging population, China has been paying more and more attention to people's health. In the report of the 19th National Congress, China puts forward the strategy of “Health China 2030,” and with the promotion of this strategic layout, the health medicine in China has been developed rapidly. Music therapy is a systematic intervention in which the therapist uses various forms of musical experiences, developed over the course of the therapy, as the driving force of the therapeutic relationship to help the client achieve wellness. The development of the discipline of music therapy began in the 1940s when the first music therapy program was established at Michigan State University in the United States. Since then, music therapy associations have been established in Canada, England, Japan, Germany, Italy, Singapore, and other countries, and music therapy has developed rapidly [1]. Currently, music therapy is relatively mature in foreign countries. Music therapy in China began in the 1980s, and although it started late, it is now being used and developed in a variety of fields.

Compared with individual therapy, group music therapy has the advantages of convenience, high acceptance, low cost, and noninvasiveness and is therefore widely used in the public health field and has achieved good results. However, group music therapy still faces some problems and challenges. First, the duration and frequency of music therapy vary widely from one to multiple sessions. The optimal duration of therapy for different conditions has not been explored. Determining the optimal dose of intervention for music therapy is an area that warrants further research. Second, previous studies have rarely assessed patients' musical experiences and preferences and taken them into account in treatment planning. This may have an impact on treatment outcomes. Therefore, treatment protocols need to be adjusted to take into account the client's preferences in the selection of repertoire in conjunction with the musical assessment of the client. Third, most studies have examined the short-term efficacy of group music therapy before and after interventions, but due to human and material constraints, long-term follow-up has not been conducted to determine its long-term efficacy [2]. Therefore, longitudinal data collection is needed. Finally, group music therapy lacks a comprehensive, unified, and scientific evaluation tool, and there are few studies on evaluation indicators.

In light of the above problems, this study introduces a new evaluation method—blockchain technology. Blockchain is the innovative power of new generation information technology and an important breakthrough for China's independent innovation of core technology. It is also included in the 14th Five-Year Plan of National Economy and has become one of the key industries of digital economy. With the development of blockchain technology and economy, the demand for data circulation and application synergy between blockchains is becoming more and more obvious. Cross-chain technology undertakes not only the transfer of data but also connects the collaboration networks behind different blockchain networks and cross-agency information exchange processes, improves the efficiency of collaboration between interrelated information modules on different blockchains, and provides technical support for the evaluation of multiple information sources. The development of blockchain cross-chain technology has formed two models, single-chain cross-chain and multichain cross-chain, and is developing into a multilevel multichain cross-chain blockchain. Importantly, the emergence of cross-chain data transfer in blockchain provides the technical conditions for two-way information collection of music performing arts and public health and also provides the methodological basis for comprehensive evaluation of the effectiveness of the application of music performing arts in the field of public health. However, most of the current studies focus on the evaluation of the impact of music on physical and mental health at the individual level, and few focus on the evaluation of music performing arts activities in the field of public health, and the evaluation methods are relatively single and lacking in science, thus hindering the potential application of music performing arts in the field of public health and limiting the development of public health-related policies.

Therefore, based on a systematic review of the relationship between music and public health, this study incorporates blockchain technology into the evaluation of the effects of music performing arts to provide a scientific evaluation of the effectiveness of music performing arts on public health and provide a relevant theoretical basis for the formulation of public health policies.

## 2. Literature Review

### 2.1. Music and Public Health: Music Therapy

Music therapy is a therapeutic technique in which the therapist uses music as a medium and applies the unique physiological and psychological effects of music to achieve the elimination of psychological barriers and the restoration or enhancement of physical and mental health through various specially designed musical behaviors, musical experiences, and musical experiences. It can be divided into individual therapy and group therapy, and in terms of techniques, it can be divided into active, passive, improvisation, and song writing. Among them, active music therapy refers to the use of singing and breathing adjustment to improve physiological indicators of the elderly, or to improve interpersonal communication, enhance the enjoyment of life, and change the state of mind through choral singing and instrument playing. Passive music therapy is an intervention that involves listening to appropriate music, accompanied by progressive muscle relaxation training, guided relaxation exercises, and song discussions to regulate the body and mind [3]. There is no significant difference in the effectiveness of active and passive music therapy in various groups, and studies have generally used a combination of active and passive interventions. The songs themselves reflect the richness of the listener's life and emotional experiences, so the music should be selected based on the age, experience, personality, and temperament of the client. Appropriate form and content can increase the homogeneity of the group members and effectively enhance the effectiveness of the group intervention.

Music therapy approaches have evolved in a variety of ways. These approaches can be broadly classified into four types: receptive music therapy, recreative music therapy, creative music therapy, and improvisational music therapy [4]. Different approaches to music therapy include a variety of different techniques. Listening is a common form of receptive music therapy, in which listening to music evokes different feelings and experiences in the client. The music therapist works in a planned and goal-oriented way through different musical experiences. Recreative music therapy invites clients to participate in specific activities that combine music with dance, singing, and games and is often used in group settings to provide opportunities for social interaction and to stimulate creativity among members. Creative music therapy is the creation of vocal or instrumental music with the client. Music composition is used as a vehicle for expressing the full range of emotions. Improvisational music therapy involves improvising with musical instruments such as mallets, string bells, triangles, tambourines, and Cajon drums. This approach does not require the client's skills to play the instrument, but rather to express emotions through the instrument, with the therapist intervening accordingly [5].

Music therapy can be divided into two types of therapy: group and individual. Group music therapy has unique advantages over individual music therapy. It creates a network of relationships between the therapist and the client and between group members, which improves the client's behavioral problems and builds the skills necessary for social integration [6]. Cohesiveness and member support play an important role in the reticulation of group music therapy. Group music therapy emphasizes a multidimensional collective interaction among the group members, interspersing playing, talking, and listening, using music and language as a vehicle for communication, and establishing a channel for expressing oneself and connecting with others in a better way, allowing for more dynamic and creative group members [7]. With music, group members are able to feel their own emotions and states in group activities, and with the facilitation of music, group members are more likely to discover the effects of their own states on themselves [8]. The discovery of one's own negative emotional experiences through others, with peer support, can also reduce participants' feelings of isolation and be more conducive to dissipating their negative internal emotions.

Group music therapy has been increasingly used in the management of anxiety in healthy, subhealthy, and ill populations to promote mental, physical, and spiritual health. Group music therapy is relatively well established abroad, having been studied in different populations such as college students, parents of premature infants with Alzheimer's disease, preoperative patients, and infertility patients [9, 10] and has been shown to be effective in improving anxiety states. In recent years, scholars have also gradually carried out the application of group music therapy in various groups of people with negative emotions such as anxiety. However, most of the studies have been conducted with dysregulated groups, especially cancer patients, psychiatric patients, and special populations [11, 12]. In conclusion, group music therapy is effective for interventions with physically and mentally challenged groups. With the development of group music therapy in the field of alleviating negative emotions such as anxiety, research has become more extensive and has begun to focus on the role of music therapy in public health [13], but fewer studies have addressed the evaluation of the role of music performing arts in public health.

Currently, the effectiveness of group music therapy in the management of negative emotions is mostly evaluated using relevant negative emotion scales before and after the intervention and the music therapist's subjective evaluation of the whole treatment process, but there are few scales to evaluate the quality of the music therapy process itself, and there is a lack of effective evaluation tools to consistently assess the music therapy process.

### 2.2. Blockchain: A New Approach to Evaluation

As an emerging Internet technology, blockchain is a decentralized, trustless distributed data ledger that has attracted widespread attention both domestically and internationally. Blockchain has been hailed as the most disruptive and innovative technology in the Fourth Industrial Revolution. China has also proposed to make blockchain an important breakthrough for autonomous innovation of core technologies. Thousands of blockchain applications have already started to be implemented, bringing not only great social and economic benefits but also playing a key role in promoting the digitization of the real economy, building a new smart city, and promoting supply-side reform [14].

The data structure of a blockchain is shown in Figure 1. From the blockchain perspective, a block is an atomic structure in the chain that records all the data in the chain, and blocks are linked to blocks to form a one-way chain structure. The consensus mechanisms used in a blockchain may be the same or different, which distinguishes the blockchain as homogeneous or heterogeneous with the block data structure. Some consensus mechanisms may appear to fork multiple chains, but in the end, the consensus mechanism can be used to determine the only master chain.

While the scale of blockchain application transactions is growing, performance bottlenecks and silos in blockchain are beginning to emerge. Firstly, the design and technical limitations of some blockchains lead to low system throughput and slow processing efficiency and large performance differences between blockchains. Secondly, the inability to quickly interoperate between different chains to meet the demand for business collaboration and data/value flows between different blockchain applications has led to the emergence of blockchain silos [15]. These issues are limiting the large-scale use of blockchain in society and industry.

Cross-chain technology is an important technical approach to achieve interconnection and interoperability of blockchain to enhance scalability and interoperability, which can solve the problems encountered in the abovementioned blockchain. In recent years, cross-chain technology has been developing rapidly, and the current mainstream cross-chain technology solutions include hash locking, notary mechanism, side chaining/relaying, and distributed keying. On the basis of these technologies, a complete cross-chain implementation solution is developed, taking into account issues such as data transfer performance, privacy and security, originality, and transaction [16]. New cross-chain solutions are constantly being proposed by blockchain platforms to solve the problems of blockchain performance bottlenecks and information silos [17].

There are currently dozens of hundreds of cross-link implementations available for users to choose from, but there are no well-developed standards for evaluating cross-link approaches. When choosing a cross-link solution, users consider a variety of factors, such as data transfer performance, privacy and security, and atomic and transactional issues. The better the data transfer performance, the more efficient the cross-link solution will be, and the more time-critical functions it will perform. Data transfer performance measurement is one of the ways to measure the data transfer performance of a solution [18]. Through data transfer performance measurement of cross-link solutions, users can obtain performance indicators of cross-link solutions, such as time delay and spit volume, and compare the data transfer performance of different cross-link solutions to facilitate the evolution and development of cross-link solutions.

### 2.3. Cross-Chain: Objective and Technology

Cross-chaining enables not only the exchange of information but also the exchange of value. This requires cross-chain to ensure both accurate two-way value circulation and accurate information flow. There are two main purposes of cross-chain: firstly, cross-chain interoperability. In blockchain system, the data on the chain can only circulate in this blockchain and cannot form a circulation with the external world, but the actual scenario often occurs in multiple chains for information exchange, which needs to enable two or more chains to change the corresponding account status and data according to a unified agreement, forming a standard cross-chain interoperability [19]. Secondly, in performance bottleneck, some blockchains have lower performance because they use some consensus mechanisms and block rules with lower performance, which limits the operation speed of blockchain and the development of blockchain ecology, resulting in the information exchange speed of blockchain system being much lower than that of traditional centralized system, and the information exchange process can be transferred to other blockchains with better performance through cross-chain technology to improve the operation of blockchain system efficiency [20].

The basis for cross-chain interoperability between blockchains is the cross-chain communication protocol, and the design of cross-chain information exchange and other functions is based on the realization of cross-chain communication. The first is the cross-chain communication protocol. The cross-chain communication needs to encapsulate the cross-chain data format, input and output interfaces, etc., and realize the transmission of block data and status information between several different blockchain networks, including the chain identifier of the source chain, the communication address of the current chain height, and the communication packet containing the starting chain identifier, the target chain identifier, the communication status, the communication survival time, and the trigger communication transaction, using relay [21, 22]. The cross-chain communication structure is implemented as shown in Figure 2. Cross-chain routing implements the interconnection topology description of multi-blockchain networks and the addressing method between blockchains based on the cross-chain communication.

Secondly, cross-chain asset exchange is one of the important directions of current cross-chain research, which aims to establish asset transfer methods between different blockchains, enabling users of different cryptographic assets to exchange assets between source and target blockchains in an atomic and trustless manner. Since it is difficult to fully replicate the state of a blockchain in another blockchain, efficient mechanisms are needed to allow the verification of events that occur on one blockchain from another blockchain without relying on the other blockchain [23]. Cross-chain atomic swapping was one of the earliest implementations, as shown in Figure 3, that could not transfer information from one blockchain to another, i.e., destroy a certain amount of information on the source blockchain and recreate the same amount of information on the target blockchain [24]. Therefore, atomic swaps always require a transaction partner willing to exchange information and thus require cross-chain platforms to provide an aggregation mechanism for information exchange partners.

Atomic exchange protocols require methods to scale to more than two users [25], as well as optimal methods to match users seeking to perform atomic exchanges, and need to enable information exchange between more blockchain users while ensuring that the total amount of assets across blockchains remains constant. Notary-based oversight of cross-chain asset exchanges is a primary approach, and the atomic cross-chain exchange protocol [26] uses third-party notaries with rewarding incentives to migrate information across blockchain ecosystems and ultimately guarantee the ultimate consistency of information standards across blockchains. Relay-based approaches are new approaches to enable cross-chain asset transfers [27], which improve relaying by applying a content-addressable storage model that enables cross-blockchain information transfer through smart contracts, where each invocation is implicitly recorded in the blockchain's information exchange history and the client can extract block header information from the information exchange history, which can be used by the relay contract to execute transactions and ensure that the provided information is actually available to the exchange's properties. The relay contract can use this information to perform transactions to ensure that the information provided can indeed be verified by the blockhead to which the exchange belongs. The convergence of multiple approaches is also a new direction, requiring the construction of a new approach to complex distributed computing to manage information assets in an adversarial environment, with the emergence of convergent approaches such as time-locked protocols and protocols that blend classical atomic protocols with modern atomic exchanges [28]. The CBC protocol, which combines classical atomic protocols and modern atomic exchanges, enables information exchange through an authenticated blockchain [29].

However, there are few studies on cross-link performance data transfer, mainly on the performance evaluation of individual cross-link solutions. The lack of generalized cross-chain data transfer performance has hindered the use and development of cross-chain solutions in blockchain platforms. In this study, we analyze the current situation and needs of cross-link solutions in blockchain platform, study the key technologies involved in each link of blockchain, propose an index system and method for evaluating the data transmission performance of cross-link solutions, and design and implement an evaluation system to evaluate the existing cross-link solutions in the industry. The feasibility and validity of the method and system are demonstrated.

## 3. Methodology

The comprehensive trust evaluation scheme proposed in this study uses cross-chain in blockchain technology to ensure the trustworthiness of static data and solve the cold start problem [30]. The static and dynamic evaluation steps are the same, but the reference data for calculation are different; i.e., the static evaluation refers to the data provided by the information provider, and the dynamic evaluation is based on the data monitored by the information after invocation. The steps of comprehensive evaluation are as follows.

**Step 1 .**

Ensure the Trustworthiness of Information. When releasing services, service providers consider that some parameters may fluctuate due to network fluctuations, causing large uncertainties, and to ensure the authenticity of the parameters, they do not adopt the simple averaging method, but set the parameters in the form of interval numbers. In the cross-chain, only the services that reach consensus can be put on the chain, and the consensus stage mainly verifies whether the parameters of information exchange are reasonable. Considering the storage performance on the blockchain, this study represents the static parameters of each service in an array, hashes the array, and stores the hash value on the block, to prevent the information from being tampered and reduce the storage pressure on the block.

**Step 2 .**

Determine the Information Requirements. The platform coarsely selects the candidate services through the user's functional requirements. Considering that different users have different requirements for the same information, the platform allows the user to set the number of intervals for the requirements of various parameters and additionally sets the maximum tolerance threshold for the negative type parameters. The threshold is set to take into account the dynamic nature of the service being invoked, and if the current dynamic information is monitored to exceed the user threshold, the appropriate service is reselected.

**Step 3 .**

The candidate information is filtered by the interval number model, and the probability of the interval number is calculated and a probability matrix is constructed. The user requirements are compared with each parameter interval provided by the service provider, and the services with intersection between the number of intervals of user requirements and the number of intervals of service release are selected. The probability matrix is then constructed by calculating the probability of the interval number. The interval number is used to take into account the dynamic variability of the service, while the likelihood is quoted to measure the degree of fit between the current service and the user's information needs.

Let any two interval numbers be *a* = [*a*^−^, *a*^*+*^], *b* = [*b*^−^, *b*^*+*^], *l*_*a*_ = *a*^*+*^ − *a*^−^, and *l*_*b*_ = *b*^*+*^ − *b*^−^. Then, the degree of possibility that *a* is greater than *b* is as follows:

(1) $$\begin{array}{c} P\left(a\geq b\right)=\max\left\{1-\max\left(\frac{b^{+}-a^{-}}{I_{a}+I_{a}},0\right),0\right\}. \end{array}$$

Considering that throughput and success rate are positive indicators and response time, cost, and latency are negative indicators in this study, the values of different indicators are represented as follows.

(2) $$\begin{array}{c} P_{ij}=\left\{\begin{array}{c} p\left(c_{ij}\geq d_{ij}\right),\\ p\left(d_{ij}\leq c_{ij}\right), \end{array}\right) \end{array}$$

where *c*_*ij*_ represents the matrix of the number of intervals of user requirements, i.e., the *j*_th_ indicator of the *i*_th_ information needs; *d*_*ij*_ represents the matrix of the number of intervals of information.

**Step 4 .**

Weight Setting. Weights are important parameters for evaluating multi-attribute questions, and traditional entropy weight method is influenced by sample data and may not match the realistic perception, while the hierarchical analysis method [31] relies too much on subjective emotion. Therefore, this study first uses the hierarchical analysis method to set the subjective weights, then uses the entropy weighting method [32] to set the objective weights and reduce the influence of subjective judgment on the weights, and finally combines the two to obtain the mixed weights.

The expert establishes the hierarchical analysis judgment matrix *f*_*ij*_ using the two-by-two comparison method on a scale of 1–9 and then verifies the matrix according to (3) and (4), where *n* is the matrix order and is the maximum *ϕ*_max_ eigenvalue of the matrix. The value of *R*_*RI*_ can be obtained from the table, and the matrix is considered valid when *C*_*CR*_ < 0.1. After passing the validation, the subjective weights are calculated from (5). The subjective weights do not change due to the change in parameters, while the objective weights change according to the static data or dynamic data. The entropy of the *ϕ*_th_ index is first calculated by equation (6) based on the probability obtained in Step 3, then the weights are calculated by equation (7), and finally the mixed weights are calculated by equation (8).

(3) $$\begin{array}{c} C_{ci}=\frac{\phi_{\max}-n}{n-1}, \end{array}$$

(4) $$\begin{array}{c} C_{cr}=\frac{C_{c1}}{R_{R1}}, \end{array}$$

(5) $$\begin{array}{c} w_{j}^{s}=\frac{\sqrt[{m}]{f_{i1}\times f_{i2}\times ...\times f_{im}}}{\sum_{j=1}^{m}\sqrt[{m}]{f_{i1}\times f_{i2}\times ...\times f_{im}}}, \end{array}$$

(6) $$\begin{array}{c} e_{j}=\frac{1}{\ln\;\;n}\sum_{i=1}^{n}P_{ij}\ln\frac{1}{P_{ij}}, \end{array}$$

(7) $$\begin{array}{c} w_{j}^{o}=\frac{1-e_{j}}{\sum_{j=1}^{m}1-e_{j}}, \end{array}$$

(8) $$\begin{array}{c} w_{j}=\gamma w_{j}^{s}+\left(1-\gamma \right)w_{j}^{o},p=1,2,...,m. \end{array}$$

**Step 5 .**

Comprehensive Service Evaluation and Ranking. The approximate ideal solution ranking method [33, 34] evaluates the services by calculating the distance between the candidate information needs and the best and worst information needs, respectively.

Firstly, according to the possible readings of the interval number in Step 3, the evaluation matrix *P* of the possible degree is established, and then, according to the corresponding mixed weights in Step 4, the weight matrix *W* is established and rewritten in diagonal form, and then, the comprehensive evaluation matrix *Z* is obtained. Then, the maximum value in each index is taken to form a positive ideal solution [35], and the minimum value in each index forms a negative ideal solution, and each candidate information service is calculated once by equations (9) to (11). Finally, the information needs that are closer to the positive ideal solution and farther from the negative ideal solution are the best information need.

(9) $$\begin{array}{c} V_{i}^{+}=\sqrt{\sum_{j=1}^{m}{\left(z_{ij}-z_{j}^{+}\right)}^{2},} \end{array}$$

(10) $$\begin{array}{c} V_{i}^{-}=\sqrt{\sum_{j=1}^{m}{\left(z_{ij}-z_{j}^{-}\right)}^{2},} \end{array}$$

(11) $$\begin{array}{c} C_{i}=\frac{V_{i}^{-}}{V_{i}^{+}+V_{i}^{-}}. \end{array}$$

Considering the cold start problem, when the information service has no history of being invoked, the evaluation is based on the static information provided by the information provider, and the evaluation level is relatively high because the information is stored in the blockchain. As the number of invocations of the information needs increases, the static weight will be from up to down, and the comprehensive evaluation of the information exchange and need should focus on the dynamic evaluation data of the current information service, so the comprehensive evaluation value of the information exchange and need is calculated as follows:

(12) $$\begin{array}{c} Q=\frac{1}{\mu +1}C_{\text{static}}+\frac{\mu }{\mu +1}C_{\text{dynamic}}. \end{array}$$

The comprehensive evaluation process is shown in Figure 4.

## 4. Discussion and Results

To validate the evaluation scheme proposed in this study, the Dataset (2.0), which was updated at the end of 2019, is used. The dataset contains 2,507 real performance metric values of Web service invocations. The performance metrics are response time (RT), throughput (TP), success rate (SA), price (BP), and latency (LC), with response time, price, and latency as negative metrics and throughput and success rate as positive metrics.

Since the newly released service has no runtime data, the static trust evaluation is weighted as 1. After each service is invoked once, the dynamic information is calculated based on the data at the time of invocation, and the comprehensive trust value is finally calculated to provide reference for subsequent user selection. As can be seen from Figure 5, the ranking of the services fluctuates slightly with the addition of real-time dynamic information when the services are invoked, which is due to the instability of information, but reflects the performance of the recently invoked information, and finally, the two are combined to make the evaluation results trustworthy and consistent with the facts. As can be seen, CSP7, CSP8, and CSP11 are no longer involved in the ranking because the subscriber sets the threshold and the most recently invoked service detected that the dynamic parameters of the services provided by these three cloud service providers exceeded the maximum tolerance threshold, so they are not included in the recommendation list.

The original static information is guaranteed to remain unchanged, but the static composite weights will change, and the change in the service ranking of the top 5 (CSP10, CSP1, CSP5, CSP13, and CSP2) is calculated as shown in Figure 6.

The degraded parameters of the first ranked service (CSP10) and the optimized parameters of the fifth ranked service (CSP2) are used to determine whether this scheme correctly reflects the change in service ranking in time (Figure 7). The static original information does not change during the experiment and *γ* = 0.5. As shown in Figure 7(a), we can see that when the QoS parameters of CSP10 and CSP2 are constantly changing, the comprehensive ranking of the service is also changing, and through continuous optimization, CSP2 changes from the worst service to the best service and CSP10 changes from the best information exchange efficiency to the worst information exchange efficiency. It is clear that the scheme in this study can correctly reflect the change in service ranking in time. In addition, the experiment observes the service ranking according to the change in user demand. With *γ* = 0.5, the service ranking of five CSPs is shown in Figure 6. As shown in Figure 7(b), it can be seen that when the user demand keeps changing, the number of intervals into which static information and dynamic information are transformed changes, and the ranking will change.

In conclusion, the comprehensive evaluation scheme proposed in this study shows good comprehensive evaluation effects in both dynamic parameter changes and information service demands, and the evaluation weights change accordingly as the number of calls increases, thus ensuring the objective and reliable evaluation results.

## 5. Conclusion

As music can nurture people's emotions and promote healthy physical and mental development, it is not difficult to conclude that music therapy is indeed very therapeutic and helpful for people's mental problems and plays a unique role in promoting people's personal development. We must not only focus on the social development of people but also on their individuality, so that they can become richer and more independent individuals. In addition to influencing people's emotions, music can also stimulate their imagination and be an effective way to subconsciously change their acceptance of certain things. Of course, music can also help people regulate their emotional problems by eliminating negative emotions, diverting their attention, calming or improving their stress and problems, evoking their inner perceptions, effectively improving their aesthetic abilities, and so on. Music is an essential part of our daily lives, and society cannot afford to be without music therapy, which is a two-pronged treatment option. Music therapy is an area worthy of further investigation and development, both from the perspective of the medical profession and from the perspective of the development of music aesthetics and the social function of music. The field of music therapy is one that is worthy of further investigation and development. More importantly, the use of group music therapy in public health is beginning to bear fruit, and music is becoming a complementary element in ensuring public health. However, few current studies have discussed comprehensive evaluation methods for public health-oriented music performing arts.

Therefore, this study proposes a dynamic comprehensive evaluation scheme based on cross-chain technology in blockchain and establishes a cross-chain-based information exchange model for the feasibility of information exchange between music performing arts and public health. The interval number model is chosen to describe static and dynamic information, respectively, for the dynamic nature of different module information, while the evaluation matrix is constructed by calculating the intervals. The subjective and objective weights are combined to set mixed weights to ensure the comprehensiveness of service evaluation.

In conclusion, this study provides technical support for the comprehensive evaluation of the effectiveness of music performing arts activities in the public health field by introducing blockchain technology while realizing the information exchange between music performing arts activities and the public health field. Given that the scheme proposed in this study is not limited to specific information modules, the method can be extended to more fields in the future.

However, it should be clarified that the technical steps of the scheme adopted in this study are still complicated, and only a small sample is adopted for the effectiveness testing session. Future research can transform the comprehensive evaluation process into a generic-only contract and enhance the practicality and generalizability of the scheme in this study by simplifying the data processing process.

## Figures and Tables

**Figure 1:** Data structure of blockchains.

**Figure 2:** Cross-chain interaction architecture based on relay.

**Figure 3:** Example of cross-chain asset atom swap process.

**Figure 4:** Comprehensive evaluation process.

**Figure 5:** Static ranking during cold start and comprehensive ranking after service call.

**Figure 6:** Influence of subjective weight importance coefficient on comprehensive service ranking.

**Figure 7:** (a) Impact of changing dynamic value on comprehensive service ranking. (b) Impact of user demand change in comprehensive service ranking.

## Data Availability

The data are available on request from the corresponding author.
